# Intracisternal administration of an interleukin-6 receptor antagonist attenuates surgery-induced cognitive impairment by inhibition of neuroinflammatory responses in aged rats

This article has been retracted.

**DOI:** 10.3892/etm.2014.2149

**Published:** 2014-12-19

**Authors:** PENG JIANG, QIONG LING, HONGBO LIU, WEIFENG TU

**Affiliations:** 1 Department of Anesthesiology, Huizhou Municipal Central Hospital, Huizhou, Guangdong 516001, P.R. China; 2 Department of Anesthesiology, Guangdong Provincial Hospital of Traditional Chinese Medicine, Guangzhou, Guangdong 510010, P.R. China; 3 Department of Anesthesiology, Guangzhou General Hospital of Guangzhou Military Command, Guangzhou, Guangdong 510010, P.R. China

**Keywords:** postoperative cognitive dysfunction, neuroinflammation, interleukin-6, aged

## Abstract

Postoperative cognitive dysfunction (POCD) is common in elderly patients, and may persist or even evolve into Alzheimer’s disease. It has been hypothesized that POCD is mediated by surgery-induced inflammatory processes. As a pro-inflammatory cytokine, the detailed role of interleukin (IL)-6 in POCD remains largely unknown. In this study, laparotomy was used to mimic human abdominal surgery in aged Sprague-Dawley rats. It was found that memory and learning were impaired following surgery, accompanied by the significant upregulation of the pro-inflammatory cytokines tumor necrosis factor α (TNF-α), IL-1β, IL-4, and IL-6. Moreover, the intracisternal administration of the IL-6 receptor (IL-6R) antagonist (tocilizumab, also know as MRA) at the time of surgery notably attenuated the surgery-induced cognitive deficit, and significantly inhibited the upregulated expression of pro-inflammatory cytokines. Further investigation indicated that the intracisternal administration of MRA inhibited the activation of the NF-κB signaling pathway in aged rats following surgery. In summary, the findings of this study suggest that IL-6 plays a crucial role in POCD, and that IL-6R antagonists may serve as novel agents for the prevention or treatment of POCD.

## Introduction

Postoperative cognitive dysfunction (POCD), commonly observed in elderly patients after surgery, is characterized by impaired concentration, memory and learning. Usually, POCD lasts days to weeks; however, it can also last longer in a small minority of patients. Advanced age is the single strongest risk factor for the development of POCD (1). In addition, accumulating evidence has shown that cardiac, abdominal and orthopedic surgeries can lead to POCD (2,3). It was originally suggested that anesthesia is a contributing factor for POCD; however, recent studies have shown no causal relationship between the depth of anesthesia and POCD (4–7). At present, POCD continues to have negative effects on the quality of life in millions of elderly patients, which brings a heavy economical burden on society. Therefore, the development of efficient strategies to prevent or treat POCD in elderly patients is urgently required.

Neuroinflammation may participate in the development of POCD, as it has been found to be involved in cognitive defects in central nervous system (CNS) diseases (8). Interleukin (IL)-6, originally identified as a B-cell differentiation factor, plays critical roles in the nervous system, and is able to activate inflammation-related signaling pathways (9–11). Moreover, the activation of signaling pathways that include nuclear factor (NF)-κB has also been demonstrated to be associated with POCD; this activation further leads to the abundant release of pro-inflammatory cytokines, including tumor necrosis factor (TNF)-α, IL-1β, IL-4, IL-6 and IL-8, and further triggers broad neuroinflammation responses in the brain (11,12). Accordingly, inhibition of the activation of pro-inflammation pathways as well as the release of pro-inflammatory cytokines appears to be a promising approach for the prevention and treatment for POCD.

In the present study, laparotomy was conducted to mimic human abdominal surgery in aged Sprague-Dawley rats, and the cognitive functions of the rats were evaluated using the Morris water maze (MWM) test. Moreover, by administering an IL-6 receptor (IL-6R) antagonist (the antibody tocilizumab, also known as MRA) at the time of surgery, the role played by IL-6 in POCD in aged rats was investigated in order to determine whether IL-6R antagonists may serve as promising agents for the prevention and treatment of POCD in elderly patients.

## Materials and methods

### Animals and groups

All protocols in this study were approved by the Ethics Committee of Huizhou Central Hospital, (Huizhou, China). Sprague-Dawley male rats (24 months old) were purchased from Hunan Environmental Biology Technical College (Changsha, China). All rats were allowed free access to clean food and water. The cage was maintained at 22±1°C on a 12 h light/dark cycle.

### Surgery

The rats were anesthetized with an intraperitoneal injection of ketamine solution (80 mg/kg) prior to laparotomy and sham surgeries. For sham-operated (control) rats (n=5), the abdominal area was shaved and cleaned with 70% ethanol, and the rats remained anesthetized for the same amount of time as the operated rats. For operated rats (n=5), a 3-cm vertical incision was made at ~0.5 cm below the lower right rib, and penetrated into the peritoneal cavity. The surgeon inserted an index finger into the opening and vigorously manipulated the viscera and musculature for 1 min. Sterile chromic gut sutures were then used to suture the peritoneal lining and muscle.

### Intracisternal administration of IL-6

To determine whether or not IL-6 plays a role in the development of POCD following surgery in aged rats, a subgroup of the operated rats (n=6) received a central administration of the IL-6R antagonist tocilizumab (MRA) (Roche Diagnostics, Basel, Switzerland) at the time of surgery. After anesthetization, the dorsal aspect of the skull was shaved and cleaned with 70% ethanol. A 27-gauge needle attached via PE50 tubing to a 25 μl Hamilton syringe was inserted into the cisterna magna. Entry into the cisterna magna was verified by drawing out 2 μl clear cerebral spinal fluid, which was then pushing back in and 3 μl MRA was administered. For vehicle controls, 3 μl sterile saline was administered.

### MWM test

On preoperative day 1 and postoperative days 3 and 7, rats were placed on the platform in the SuperMaze Morris (XR-XM101; Xinruan Co., Shanghai, China) for 30 sec, and then released into the water from an assigned release point. For each assay, rats were allowed to swim until they found and landed on the platform. If they failed within 60 sec, the rats were picked up and placed on the platform for 30 sec. This assay was repeated 5 times, and rats were allowed to stay on the platform for 30 sec between assays. Swimming distance and time were recorded using video tracking. Data were analyzed by MWM software.

### Reverse transcription-quantitative polymerase chain reaction (RT-qPCR)

The rats were sacrificed by cervical dislocation under etherization. The hippocampal tissues of the rats were minced prior to total RNA extraction using TRIzol reagent (Invitrogen Life Technologies, Carlsbad, CA, USA) according to the manufacturer’s instructions. Expression of mRNA was examined using the standard SYBR Green RT-PCR kit (Takara, Otsu, Japan), in accordance with the manufacturer’s instructions. PCR was conducted using 1 μg total RNA on an ABI 7500 thermocycler (Applied Biosyystems Life Technologies, Carlsbad, CA, USA). The PCR conditions were set at: 95°C for 10 min (initial denaturation), followed by 40 cycles of 95°C for 20 sec, 62°C for 30 sec and 72°C for 30 sec (amplification). The specific primer pairs were as follows: TNF-α, sense: 5′-CATGATCCGAGATGTGGAACTGGC -3′; antisense: 5′-CTGGCTCAGCCACTCCAGC-3′; IL-1β sense: 5′-GATGGCTGCTATTCCTAATCC-3′; antisense: 5′-ATACTGCCCATTCTCGACAAG-3′; IL-4: sense: 5′-GCT ATTGATGGGTCTCACCC-3′; antisense: 5′-CAGGACGTC AAGGTA-3′; IL-6: sense: 5′-ACTCACCTCTTCAGA ACGAATTG-3′; antisense: 5′-CCATCTTTGGAA GGTTCAGGTTG-3′; and for β-actin (as an internal reference), sense: 5′-AGGGGCCGGACTCGTCATACT-3′; antisense: 5′-GGCGGCACCACCATGTACCCT-3′. The relative expression of mRNA was quantified using 2^–ΔΔCt^ method.

### Western blotting

Protein was extracted from the hippocampal tissue of the rats using a Nuclear and Cytoplasmic Protein Extraction kit (Pierce, Thermo Scientific, Rockford, IL, USA). The protein concentration was determined by the Bradford DC protein assay (Bio-Rad, Hercules, CA, USA). The proteins were then separated in 10% SDS-PAGE and transferred onto a polyvinylidene difluoride (PVDF) membrane, which was then incubated with phosphate-buffered saline (PBS) containing 50 g/l skimmed milk at room temperature for 4 h. Then, the PVDF membrane was incubated with mouse anti-rat monoclonal NF-κB P65 (1:50 dilution) and mouse anti-rat monoclonal GAPDH (1:100 dilution) primary antibodies (Abcam, Cambridge, UK), respectively, at 37°C for 1 h. After washing with PBS three times, the PVDF membrane was incubated with the goat anti-mouse peroxidase-conjugated secondary antibody (Abcam) at room temperature for 1 h. Chemiluminescent detection was performed using an ECL kit (Pierce Chemical, Rockford, IL, USA).

### Statistical analysis

All data are expressed as the mean ± standard deviation (SD). Differences between two groups were determined by a Student’s t-test. All analyses were performed using SPSS software, version 16.0 (SPSS, Inc., Chicago, IL, USA). P<0.05 was considered to indicate a statistically significant result.

## Results

### Aged rats show defects in cognitive function following surgery

Swimming time and distance in the MWM were used to evaluate the cognitive function. On preoperative day 1 and postoperative days 3 and 7, rats were placed on the platform in the MWM for 30 sec, and then released into the water from an assigned release point. Rats were allowed to swim until they found and landed on the platform. As shown in Fig. 1, swimming time and distance were significantly increased on days 3 and 7 after surgery, when compared with those on day 1 prior to surgery. These findings indicate that the cognitive function of the rats was impaired after surgery.

### Intracisternal administration of IL-6R antagonist attenuates defects in cognitive function in aged rats following surgery

To determine whether IL-6 had an effect on cognitive function following surgery in aged rats, some of the animals received a central administration of the IL-6R antagonist MRA at the time of surgery. The effect of MRA on the surgery-induced cognitive defects in the aged rats was investigated. As shown in Fig. 2, the swimming time and distance were significantly decreased in the rats treated with MRA on days 3 and 7 after surgery, when compared with those in the control group. These findings indicate that MRA attenuated the surgery-induced cognitive defects in the aged rats, and suggest that IL-6 played a role in the development of POCD in the rats following surgery.

### Intracisternal administration of IL-6R antagonist inhibits the upregulation of pro-inflammatory cytokines in aged rats following surgery

RT-qPCR was further used to determine the mRNA levels of pro-inflammatory cytokines in the brains of the aged rats at 24 h after surgery, with or without MRA administration. Rats that received sham surgery were used as controls. As shown in Fig. 3, the mRNA expression levels of TNF-α, IL-1β, IL-4 and IL-6 were significantly upregulated 24 h after surgery, when compared with those in the control group. However, the intracisternal administration of MRA notably attenuated the surgery-induced upregulation of these pro-inflammatory cytokines. These findings suggest that blocking IL-6-mediated pro-inflammatory signaling effectively inhibits surgery-induced neuroinflammatory responses in aged rats.

### Intracisternal administration of IL-6R antagonist inhibits activation of the NF-κB signaling pathway in aged rats following surgery

The underlying molecular mechanism was further investigated. As activation of the NF-κB signaling pathway has been reported to play a crucial role in neuroinflammatory responses (13), the activity of the NF-κB pathway was determined in each group using a western blotting assay. As demonstrated in Fig. 4, the protein level of NF-κB P65 in the cell nuclei was significantly upregulated 24 h after surgery, when compared with that in the control group, and this upregulation was attenuated following the intracisternal administration of MRA. These findings suggest that the IL-6R antagonist effectively inhibited the surgery-induced activation of NF-κB signaling in the brains of aged rats.

## Discussion

As a global issue, POCD is worsening as aging of society is increasing (14). Accordingly, it is urgently necessary to identify its molecular mechanism as well as therapeutic targets. To the best of our knowledge, the present study demonstrated for the first time that blocking the IL-6R effectively inhibited surgery-induced cognitive defects in aged rats, as well as the upregulation of several key pro-inflammatory cytokines, which was at least partially achieved through suppressing the activation of NF-κB signaling.

In recent years, several factors have been demonstrated to contribute to POCD, including surgery-induced neuroinflammation (9,15). Any changes including surgery may disturb the homeostasis in the brain, which will activate microglia and lead to the secretion of pro-inflammatory factors (11,16,17). In addition, surgery also leads to the upregulation of peripheral pro-inflammatory cytokines, which can also enter the brain through the deficient areas of the blood-brain barrier and further activate microglia (8,18,19). In the present study, it was found that following surgery, pro-inflammatory cytokines were significantly upregulated in the aged rat brain. However, it has been well-established that excessive pro-inflammatory cytokines cause excessive neuroinflammation, which can contribute to POCD.

IL-6 has been reported to be involved in neurogenesis by affecting both glial cells and neurons, as well as the response of mature neurons and glial cells in normal conditions and various injury models (20). It has been reported that the expression of IL-6 is influenced in several of the main brain diseases, and IL-6 has been suggested to have a role in the observed neuropathology; therefore, it may become a promising therapeutic target (21,22). However, the detailed role of IL-6 in surgery-induced POCD in elderly patients remains largely unknown. In the present study, it was demonstrated that the expression of IL-6 was significantly upregulated following surgery, accompanied by the upregulation of other inflammatory cytokines, which is consistent with the findings by Yu *et al* that IL-6, as well as TNF-α, IL-1β and IL-8, are significantly upregulated in the hippocampal tissues of aged rats following splenectomy (23). Moreover, Hovens *et al* also revealed that abdominal surgery induced the upregulation of plasma levels of IL-6, as well as decreased cognitive flexibility, increased microglia activation and increased weight loss (24). In addition, Peng *et al* performed a meta-analysis of 13 studies, and showed that the serum concentration of IL-6 was notably upregulated in patients with POCD when compared with those without POCD, suggesting that POCD is indeed correlated with the concentration of the peripheral inflammatory marker IL-6 (25).

To further investigate the role of IL-6 in surgery-induced cognitive defects in aged rats, an IL-6R antagonist was used, and it was found that blocking the central signaling of IL-6 with a single intracisternal administration of the IL-6R antagonist at the time of surgery was sufficient to suppress surgery-induced cognitive defects, the upregulation of inflammatory cytokines, and activation of NF-κB signaling in aged rats. This indicated that the inflammatory response, particularly that mediated by IL-6 in the brain following surgery, is critical for the development of POCD in aged rats. Furthermore, the data is similar to that in a previous study reporting that blocking the IL-1 receptor using an IL-1R antagonist in the brain also inhibited surgery-induced cognitive impairments in aged rats, suggesting that these inflammatory cytokines may be used as novel preventive or therapeutic targets for POCD (26).

In addition, it has been well established that excessive activation of NF-κB signaling pathway plays a key role in the development of POCD (23). Once activated, the phosphorylation of IκBs is upregulated, and then the degradation of IκBs occurs, which promotes the nuclear translocation of NF-κB. As a key transcriptional factor, NF-κB enters into the nucleus and promotes the transcription of various genes, including pro-inflammatory cytokines such as IL-6, as well as TNF-α, IL-1β and IL-8 (27). In the present study, the protein levels of IκBa as well as those of NF-κB P65 in cell nuclei were reduced by the administration of an IL-6R antagonist during surgery, suggesting that the inhibition of IL-6 indirectly suppressed the activation of the NF-κB pathway.

In conclusion, the data revealed in the present study suggest that IL-6 contributes to surgery-induced neuroinflammation in aged rats, partially at least, via the activation of NF-κB signaling, which ultimately results in POCD. Therefore, this study identified an important role of IL-6 in the development of POCD, suggesting that the IL-6R may be used as a promising target for the prevention and treatment of POCD.

## Figures and Tables

**Figure 1:** Swimming distance and time of aged rats in the Morris water maze. Results presented are the mean ± standard deviation. Pre Day1, the Morris water maze test was performed one day prior to surgery; Post Day3, the Morris water maze test was performed on the third day after surgery; Post Day7, the Morris water maze test was performed on the seventh day after surgery. ^**^P<0.01 vs. Pre Day1.

**Figure 2:** Swimming distance and time of aged rats in the Morris water maze assay. Results presented are the mean ± standard deviation. Day3, the Morris water maze test was performed on the third day after surgery; Day7, the Morris water maze assay was performed on the seventh day after surgery; control, rats received surgery without MRA (tocilizumab); MRA, rats received surgery with MRA. ^**^P<0.01 vs. control.

**Figure 3:** Relative mRNA expression of the pro-inflammatory cytokines TNF-α, IL-1β, IL-4 and IL-8 in rat hippocampal tissues. Results presented are the mean ± standard deviation. Control, rats received sham surgery; surgery, rats received surgery without MRA (tocilizumab); surgery + MRA, rats received surgery with MRA; TNF, tumor necrosis factor; IL, interleukin. ^**^P<0.01 vs. control.

**Figure 4:** Protein expression of NF-κB P65 in cell nuclei and total cell lysate in rat hippocampal tissues. GAPDH was used as an internal reference. Results presented are the mean ± standard deviation. Control, rats received sham surgery; surgery, rats received surgery without MRA (tocilizumab); surgery + MRA, rats received surgery with MRA; NF, nuclear factor. ^**^P<0.01 vs. control.
